The article "Study on the Absorption of Arsenic Species in Realgar Based on the Form and Valence" was published in 2022. Journal: Evid Based Complement Alternat Med.

# Study on the Absorption of Arsenic Species in Realgar Based on the Form and Valence

**DOI:** 10.1155/2022/1026672

**Published:** 2022-08-23

**Authors:** Mingyi Sun, Yaolei Li, Ying Wang, Huimin Wu, Jing Liu, Longtai You, HuLinyue Peng, Huating Huang, Hongyu Jin, Xiaoxu Dong, Changhai Qu, Xingbin Yin, Jian Ni

**Affiliations:** ^1^School of Chinese Materia Medica, Beijing University of Chinese Medicine, Beijing 102488, China; ^2^Institute for Control of Chinese Traditional Medicine and Ethnic Medicine, National Institutes for Food and Drug Control, Beijing 102629, China

## Abstract

At present, several experiments have been carried out to study the changes in total arsenic content of realgar and its prescription, but few researches on its form and valence. We evaluated the change in arsenic species concentration in realgar from the perspective of absorption by using an *in vitro* dissolution study, an *in vivo* unidirectional intestinal perfusion study, transmembrane transport in Caco-2 cells, and a pharmacokinetic study in rats. In the gastrointestinal tract, arsenic species are mainly present inorganic forms of AsIII and AsV. The cumulative dissolution rates of soluble arsenic in 4 h artificial gastric fluid and 8 h artificial intestinal fluid were 21.99% and 59.20%, respectively. The *P*_app_ values of soluble arsenic in realgar in the duodenum, jejunum, and ileum of rats were 5.4 × 10^−3^, 6.1 × 10^−3^ and 5.8 × 10^−3^ cm/min, respectively. In the process of small intestine perfusion, the AsIII of realgar was partially converted into AsV in the duodenum and jejunum. As the transport time increased, the transmembrane transport rate and *P*_app_ value of soluble arsenic in realgar were increased in Caco-2 cells, and it also suggested that arsenic species may be passively transported across the Caco-2 cell monolayer. The *C*_max_ and AUC _(0-24)_ of AsIII, AsV, and DMA in plasma of realgar were 41.26 ng L^−1^/343.977 ng h mL^−1^, 21.626 ng L^−1^/47.310 ng h mL^−1^, and 2.372 ng L^−1^/30.429 ng h mL^−1^, respectively. *T*_max_ and MRT _(0-∞)_ of AsIII, AsV, and DMA were 2.571 h/9.649 h, 0.393 h/2.790 h, and 3.143 h/23.145 h, respectively. It is hoped to provide a basis for clarifying the arsenic species in realgar.

## 1. Introduction

Realgar (As_4_S_4_) has been used for more than 2000 years to treat diseases, such as carbuncles, insect and snake bites, intestinal parasitosis, tumors, leukemia, and malignant lymphoid system diseases in China [1, 2]. Chinese medicine compound preparations containing realgar have been widely used, and 37 kinds of realgar-containing Chinese patent medicines were included in the 2020 edition of the Chinese Pharmacopoeia. Realgar exhibits efficacy and toxicity *in vivo*. Arsenic, the main component of realgar, undergoes biotransformation after entering the body. Through oxidation-reduction, methylation, biosynthesis, and other processes, it can be converted into different species (Figure 1) [3, 4]. Arsenic mainly exists in the form of +3 and +5 valences in compounds. The existing forms of arsenic in the body mainly include inorganic arsenic (AsIII and AsV), organic arsenic (MMA, DMA, AsB, and AsC), and arsenic biomacromolecules (combination of different arsenic compounds with transferrin or hemoglobin) [5].  Figure 2 exhibits the chemical structures of six common arsenic species. Generally, inorganic arsenic is more toxic than organic arsenic, and the toxicity of trivalent is higher than pentavalent [6]. The activity, toxicity, bioavailability, and metabolic pathways of arsenic in the human body are closely related to its existing form. Therefore, it is very important to study the arsenic form and valence state of realgar.

Oral administration is the most widespread way for taking realgar, and the absorption in the intestine is the key factor in deciding the bioavailability of realgar and affects the therapeutic efficacy of drugs. At present, there are few studies on the gastrointestinal absorption of realgar. Thus, the aim of this work was to evaluate the absorption of arsenic in realgar by the means of utilizing an *in vitro* dissolution study, an *in vivo* unidirectional intestinal perfusion study, transmembrane transport in Caco-2 cells, and pharmacokinetic stud in rats. High-performance liquid chromatography-inductively coupled plasma-mass spectrometry (HPLC-ICP-MS) is the most commonly used method for the detection of arsenic species. Thus, we established an HPLC-ICP-MS method for the detection of six arsenic species: AsB, AsIII, AsV, MMA, DMA, and AsC. Therefore, the arsenic species of realgar in the process of absorption will be revealed.

## 2. Materials and Methods

### 2.1. Chemical and Reagents

Realgar (batch number: 212201) was purchased from Beijing Huamiao Pharmaceutical Co Ltd (Beijing, China). Standard solutions of AsB, AsIII, DMA, MMA, AsC, and AsV were purchased from the National Institute of Metrology (Beijing, China). Pepsin, trypsin, and MTT were purchased from Biotopped Science and Technology CO Ltd (Beijing, China). All other chemicals were of analytical grade. Fetal bovine serum (FBS), MEM-EBSS, NEAA, trypsin (0.25%, w/v), penicillin, and streptomycin were purchased from Gibco (Beijing, China). DMSO was purchased from Sigma (St. Louis, MO, USA). Hanks balanced salt mixture (HBSS) and phosphate buffer solution (PBS) were purchased from Corning (Corning, NY, USA). An alkaline phosphatase kit was purchased from Nanjing Jiancheng Bioengineering Research Institute (Nanjing, China). Ammonium carbonate and sodium carboxymethyl cellulose were obtained from Beijing Chemical Factory (Beijing, China). Concentrated nitric acid (70%) was purchased from Shanghai Aladdin Biochemical Technology Co Ltd (Shanghai, China). Acetonitrile was purchased from Sigma Aldrich Chemicals (MO, USA). Sodium chloride injection was obtained from Shijiazhuang No. 4 Pharmaceutical Co Ltd (Shijiazhuang, China). Krebs-Ringer (K-R) powder was obtained from Shanghai Yuanye Biotechnology Co Ltd (Shanghai, China).

### 2.2. Animals

Male Wistar rats (250 g ± 20 g) were purchased from SPF (Beijing) Biotechnology Co Ltd (Beijing, China). They lived in an environment with a humidity of (50 ± 10)% and a temperature of (25 ± 2)°C. Artificial lighting was supplied on a fixed half-day light and half-day dark cycle, with food and water available randomly. All animal procedures were approved by the Ethical Committee of Beijing University of Chinese Medicine (No. BUCM-4-2021051201-2025), according to the Guide for the Care and Use of Laboratory Animals released by the National Institutes of Health.

### 2.3. The Conditions of HPLC-ICP-MS

The ICP-MS conditions were summarized as follows: the feedback power at 5 W, the RF power at 1550 W, the flow rate of high-purity argon at 1.00 L·min^−1^, the flow rate of plasma gas at 15.0 L·min^−1^, the rotation speed of the peristaltic pump to be 0.2 rps, the detection mass number to be *m*/*z* = 75 (As), and the acquisition time to be consistent with that of the liquid phase.

The Agilent 7700 ICP-MS (Agilent Technologies, USA) equipped with an Agilent 1100 HPLC (Agilent Technologies, USA) for chromatographic separations was used to detect and quantify arsenic speciation compounds. Samples were analyzed on a Dionex Ion Pac™AS7 (4 × 250 mm, 5 *μ*m) with a flow rate of 1 mL/min. The mobile phase was 0.025 mol L^−1^ ammonium dihydrogen phosphate solution (ammonia regulating pH 8.0) (A) and ultrapure water (B), and the gradient elution program is shown in the following table (Table 1).

### 2.4. Preparation of Arsenic Species Standard Solution

Accurately transfer an appropriate volume of standard solutions of six arsenic species of AsB, AsIII, AsV, MMA, DMA, and AsC, and then, add ultrapure water to make each 1 mL containing 1 μg of each arsenic compound solution a mixed standard stock solution.

### 2.5. *In Vitro* Dissolution Study

The artificial gastric fluid was prepared with 16.4 mL of dilute hydrochloric acid, 800 mL of water, and 10 g of pepsin. After shaking, extra water was added to make the final volume to 1000 mL. The artificial intestinal fluid was prepared by adding 6.8 g potassium dihydrogen phosphate into 500 mL of water to dissolve, using a 0.1 mol·L^−1^ sodium hydroxide solution to adjust the pH value to 6.8, and preparing another solution by adding 10 g trypsin into the proper amount of water. Then, the two solutions were mixed and water was added to make up to 1000 mL.

0.083 g realgar was added to 15 mL of artificial gastric fluid and 15 mL of artificial intestinal fluid, respectively. Samples were maintained in vials at 37°C ± 2°C. Then, we stirred them with a magnetic bar at 100 rpm without light. 0.2 mL of artificial gastric dissolved medium was collected at 1, 2, and 4 hours interval, and 0.2 mL of artificial intestinal dissolved medium was collected at 2, 4, 6, and 8 hours interval. Meanwhile, 0.2 mL of fresh medium was added to the vials. The sample solutions were centrifuged at 6000 rpm for 10 min. Then the supernatants were diluted with high-purity water and filtered using a 0.45 *μ*m millipore filter membrane. HPLC-ICP-MS was used to determine the sample content.

The cumulative dissolution amount was calculated by the following equation:

(1) $$\begin{array}{c} F=C_{t}\times V_{0}+V\times \sum C_{i}, \end{array}$$

where *C*_t_ is the concentration of arsenic compounds measured at time *t*, V_0_ is the volume of dissolution medium (15 mL), V is the sampling volume (0.2 mL), *C*_i_ is the concentration of arsenic species measured before time *t*, and F is the cumulative dissolution amount at time *t*.

### 2.6. *In Vivo* Unidirectional Intestinal Perfusion Study in Rats

Considering that realgar is insoluble in perfusate, it is necessary to simulate the process from the stomach to the duodenum as much as possible. Realgar was dissolved in artificial gastric fluid and then diluted with Krebs-Ringer solution to obtain intestinal perfusate. Rats were fasted for 12 hours. The rats were anesthetized by intraperitoneal injection of 2% pentobarbital sodium. The abdominal cavity was opened along the midline of the abdomen and intubated, ligated, and fixed on both sides of the duodenum, jejunum, and ileum. Cover the wound with absorbent cotton soaked in normal saline and keep warm with infrared light. Firstly, rinse the intestine with normal saline preheated to 37°C, and pump air to flush out normal saline. Then perfuse with the test solution of known weight, fill the intestinal tract with the drug solution at a high flow rate, reduce the flow rate to 0.25 mL/min, discard the perfusion solution for 30 min, and then quickly replace the vial containing the test solution of known weight and the vial collecting the perfusion solution of known weight every 15 min. Calculate the weight of the test solution pumped in and the weight of the perfusion solution collected every 15 minutes. Finally, the length and circumference of the intestinal segment were measured. Take the perfusion solution, vortex for 1 min, centrifuge at a high speed (10000 r/min, 10 min), and analyze the supernatants using HPLC-ICP-MS.

The absorption rate constant (*K*_a_) and apparent permeability coefficient (*P*_app_) were calculated by the following equation:

(2) $$\begin{array}{c} K_{a}=\left(1-\frac{C_{\text{out}}V_{\text{out}}}{C_{\text{in}}V_{\text{in}}}\right)\times \frac{Q}{V}, \end{array}$$

(3) $$\begin{array}{c} P_{\text{app}}=-Q\frac{\text{ln}\left(C_{\text{out}}V_{\text{out}}/C_{\text{in}}V_{\text{in}}\right)}{2\pi rl}, \end{array}$$

where *C*_in_ and *C*_out_ are the concentrations of the perfusate at the inlet and outlet (ng/mL), respectively, *V*_in_ and *V*_out_ are the volumes of the test solution injected and collected, respectively (corrected by the gravimetric method, assuming the same density of the solutions at the inlet and outlet), *Q* is the perfusion velocity (0.25 mL/min), V = *πr*^*2*^*L* is the volume of the perfused intestinal segment (cm^3^), and *r* and *l* are the radius (cm) and length (cm) of the perfused intestinal segment, respectively.

The soluble arsenic absorption rate was calculated by following the equation:

(4) $$\begin{array}{c} \text{Absorption rate}\left(\%\right)=\left(1-\frac{\sum C_{\text{out}}V_{\text{out}}}{\sum C_{\text{in}}V_{\text{in}}}\right)\times 100\%. \end{array}$$

### 2.7. Transmembrane Transport in Caco-2 Cells

#### 2.7.1. Cell Culture

Caco-2 cells were purchased from the National Infrastructure of Cell Line Resources (3111C0001CCC000100, Beijing, China). Caco-2 cells were cultured in MEM supplemented with 20% FBS, 1% NEAA, and 1% penicillin and streptomycin. The cells were grown in an atmosphere of 5% CO_2_ and 95% relative humidity at 37°C. The medium was changed every 2-3 days. After reaching 80%–90% confluence, the cells were subcultured with 0.25% trypsin. In this research, cells between 30 and 40 passages were chosen.

#### 2.7.2. Cytotoxic Effects of Drug Dissolutions in Caco-2 Cells

Cell viability was examined by the MTT assay to select the concentrations to be used in the next step. The Caco-2 cells (1 × 10^4^ cells/well) were plated into 96-well plates. After 24 h, the cells were incubated with a series of concentrations of realgar artificial intestinal dissolved solution (RI) *in vitro* (diluted 10, 20, 50, 100, 200, 500, and 1000 folds, respectively). The cells of the control group were cultured in MEM medium. After 24 hours of incubation, both cells in the control group and the treated group were cultured in 0.5 mg/mL MTT solution for 4 h at 37°C, followed by the removal of MTT medium. The resultant formazan crystals were dissolved in 150 *μ*L DMSO. The 96-well plates were shaken for 5 min and measured at 490 nm using an automatic microplate reader (Thermo, Multiskan GO, USA). The relative viability of the cells in the treated group was expressed as percentage of the cells in the control group.

#### 2.7.3. Cell Transport Tests

Monolayer integrity was assessed before the transport test. Thus, transepithelial electrical resistance (TEER) was measured by Millicell-ERS (Millipore Corporation, Billerica, MA, USA), and the alkaline phosphatase (AKP) activity was determined. During the growth and differentiation of the cultures on the transwell membranes, TEER should be measured every 2-3 days, and AKP activity were detected 3-4 times by using the AKP kit.

Caco-2 cells were plated at a density of 2 × 10^5^ cells/mL on the polyester membranes in transwell chambers. The medium was changed every 1-2 days until monolayers were formed. Before the transport tests, the cells were washed with 37°C HBSS three times and then incubated at 37°C for 20 min. 0.5 mL of drug-dissolved solution was added on the apical side (A side), and 1.5 mL of HBSS was added on the basolateral side (B side) to test the transport from A to B sides. At the stipulated test times (30, 60, 90, 120, and 180 min), 600 *μ*L samples were taken from the B side and replaced with the same volume of the new medium. Samples were centrifuged at 10,000 rpm for 10 minutes at 4°C. The supernatants were analyzed using HPLC-ICP-MS.

The transmembrane transport rate and apparent permeability coefficient (*P*_app_) were calculated by the following equation:

(5) $$\begin{array}{c} \text{Transmembrane transport rate}\left(\text{\%}\right)\;=\frac{\text{Cumulative transport amount}}{\text{Initial quality of sample}}\times 100\text{\%,} \end{array}$$

(6) $$\begin{array}{c} P_{\text{app}}=\frac{dQ/dt}{AC}, \end{array}$$

where dQ/dt represents the apparent appearance rate of arsenic speciation in the receiver side; A represents the surface area of monolayers, 1.12 cm^2^; and C represents the initial arsenic concentration in the donor side.

### 2.8. Pharmacokinetic Study

Realgar was mixed with 0.5% (w/v) sodium carboxymethylcellulose. Rats were fasted for 12 hours. Six rats were orally dosed with 0.1 g/kg of realgar after seven days of acclimation. The blood (about 0.4 mL) from the ocular fundus veins of rats was collected into heparinized polythene tubes at 0, 0.083, 0.25, 0.5, 0.75, 1, 2, 4, 8, 12, and 24 hours after the oral administration, and the plasma was separated by centrifugation at 4000 rpm for 10 min and stored at −80°C before analysis. Plasma samples were thawed to room temperature before use. 300 *μ*L acetonitrile was added into a 100 *μ*L plasma sample for protein precipitation. The mixture was centrifuged at 12000 rpm for 10 min at 4°C after vortex-mixing for 1 min. The supernatant was dried under nitrogen and dissolved in 100 *μ*L of water. The mixture was centrifuged at 10000 rpm for 10 min at 4°C. The resulting supernatant was analyzed using HPLC-ICP-MS. The pharmacokinetic parameters including the area under the concentration-time curve (AUC), peak plasma concentration (*C*_max_), elimination half-life (*t*_1/2_), and mean residence time (MRT) of the arsenicals were calculated by the noncompartmental analysis using the DAS version 3.0 program.

### 2.9. Statistical Analysis

The methods of statistical analyses were one-way ANOVA and Dunnett's multiple comparison tests for multiple comparisons using SPSS version 17 software (SPSS Company, Chicago, IL, USA). *P* < 0.05 was considered statistically significant.

## 3. Results and Discussion

### 3.1. Analytical Method Validation

The retention times of AsB, AsIII, DMA, MMA, AsC, and AsV were 1.5, 1.8, 3.7, 5.8, 7.5, and 16.3 min, respectively. The linear ranges for AsB, AsIII, DMA, MMA, and AsC were all between 1 and 300 ng/mL with linear coefficients greater than 0.9997, and the detection limits were 1 ng/mL. AsV had good linearity in the range of 2.5 ng/mL∼300 ng/mL with a linear coefficient of 1.0000. The LLOQ was 2.5 ng/mL for AsV. The intra- and interday accuracy and precision were determined by QC samples at low (2.5 ng/mL), medium (20 ng/mL), and high concentrations (200 ng/mL). The intra- and interday precision (RSD%) was lower than 6.89%. The matrix effect RSD of the six arsenic species is less than 8.55%, and the recovery RSD values are less than 12.35%. The stability of AsB, AsIII, DMA, MMA, AsC, and AsV under different storage conditions was measured. Stability study results showed that six species were stable at 4°C for 24 h, three freeze-thaw cycles, and −20°C for one month. The above results indicate that this method could be used for arsenic species analysis of Realgar and its compound.

### 3.2. *In Vitro* Dissolution Study

The pH of human gastric fluid is between 1 and 4 (differences between fasting and food). In general, it takes about 3 to 4 hours for the stomach to empty completely [7]. The small intestine is the main site of absorption. The pH value of the small intestinal fluid is between 5 and 7, and the food stays in the small intestine for 3 to 8 hours [7]. Therefore, the dissolution within 4 hours in artificial gastric fluid and the dissolution within 8 hours in the artificial intestinal fluid were investigated.

The cumulative dissolution results are shown in Figure 3. In this study, we detected two arsenic compounds, AsIII and AsV, which are inorganic arsenic forms. It is consistent with the study that soluble arsenic mainly exists in the gastrointestinal fluid in the inorganic form of AsIII and AsV [8]. Soluble arsenic is the sum of AsIII and AsV. In artificial gastric fluid, the cumulative dissolution amount of AsIII and AsV in realgar increased with the increase of dissolution time within 0∼4 h. In the artificial intestinal fluid, the AsIII in realgar increased with the increase in the dissolution time within 0∼8 h. The dissolution of AsV decreased a little over time after 2 h. We speculated the reason may be that AsV in realgar was almost completely dissolved at 2 h, but as the dissolution time increased, a little AsV adhered to the surface of the realgar powder, and the content of AsV in the solution decreased slightly.

From the results in Figure 4, the dissolution of AsIII and soluble arsenic in realgar was significantly higher than that in artificial gastric fluid at 2 h and 4 h (*P* < 0.05), and the dissolution of AsV in artificial intestinal fluid at 2 h was significantly higher than that in artificial gastric fluid (*P* < 0.05). It showed that the dissolution of inorganic arsenic species varies greatly in different pH environments. AsIII is a polyhydroxy inorganic weak acid with a pKa value of 9.2. The pKa of AsV is 2.3, 6.8, and 11.3, and it mostly exists in the form of H_2_AsO_4_^−^ and/or HAsO_4_^2-^ [9]. The pH of artificial gastric fluid is 1.2, and the pH of artificial intestinal fluid is 6.8 [10]. Therefore, the dissolved amount of arsenic in artificial intestinal fluid was more than that in the artificial gastric fluid in the same period.

By comparing the cumulative dissolution rate of realgar in artificial gastrointestinal fluid, the dissolution degree of soluble arsenic in different times and media was discussed. The cumulative dissolution rate of soluble arsenic in the artificial gastric fluid reached 21.99% in 4 h, and the cumulative dissolution rate of soluble arsenic in the artificial intestinal fluid was 59.20% at 8 h (Table 2).

### 3.3. *In Vivo* Unidirectional Intestinal Perfusion Study in Rats

In the *in vivo* unidirectional intestinal perfusion experiment in rats, two inorganic forms of arsenic, AsIII and AsV, were mainly detected, and they were detected in the duodenum, jejunum, and ileum. The chromatographic peaks of MMA and DMA appeared in intestinal perfusate samples, but could not be quantitatively analyzed due to the low content. Therefore, the results mainly show the concentration ratios of AsIII, AsV, and soluble arsenic (the sum of AsIII and AsV) before and after perfusion, as well as intestinal absorption parameters.

#### 3.3.1. Concentration Ratio of Arsenic Species before and after Perfusion

*C*_in_ and *C*_out_ are the concentrations of arsenic species in the inlet and outlet perfusates, respectively. By comparing the concentration of perfusate before and after intestinal perfusion in rats, information on the absorption changes of arsenic species in different intestinal segments and at different times was obtained. When *C*_out_/*C*_in_ < 1, the outlet perfusate concentration was lower than the inlet concentration, the drug was absorbed in the intestinal segment, and the concentration decreased. When C_out_/*C*_in_ >1, the concentration of the outlet perfusate was higher than that of the inlet, and the drug concentration increased, suggesting that new components may be transformed.

As shown in Table 3, in the duodenum and jejunum, *C*_out_/*C*_in_ results of AsV >1, the AsV concentration increases after intestinal perfusion, indicating that new AsV was generated. *C*_out_/*C*_in_ results of AsIII <1, the concentration of AsIII decreased after perfusion, indicating that AsIII was absorbed in the duodenum and jejunum, and part of AsIII was converted into AsV, which increased the concentration of AsV after perfusion. In the ileum, *C*_out_/*C*_in_ results of AsIII and AsV <1, and both components were absorbed. In terms of soluble arsenic, *C*_out_/*C*_in_ < 1, arsenic in the realgar intestinal perfusate was absorbed in the duodenum, jejunum, and ileum. Comparing the three intestinal segments, the *C*_out_/*C*_in_ values of AsIII and soluble arsenic were duodenum < jejunum < ileum, and the *C*_out_/*C*_in_ value of AsV was duodenum > jejunum > ileum, suggesting that in the realgar perfusate the absorption or biotransformation of arsenic species was higher in the duodenum than in the jejunum and ileum. There were differences in absorption and transformation capacity in different intestinal segments.

From the above results, it can be found that arsenic species not only have an absorption process but also a biotransformation process in the small intestine. There are differences in the absorption and transformation capacity of arsenic species in different intestinal segments. The small intestine can not only absorb drugs but also metabolize drugs. It is one of the main parts of drug metabolism in addition to the liver. Therefore, after the intestinal perfusate passed through the small intestine of rats, a part of AsIII in realgar was converted into AsV.

#### 3.3.2. The Absorption Rate Constant (*K*_a_), Apparent Permeability Coefficient (*P*_app_), and Absorption Rate of Soluble Arsenic in the Small Intestine

Because the realgar intestinal perfusate passes through the duodenum and jejunum, a part of AsIII is converted into AsV, the concentration of AsV is higher than the initial concentration, and the values of *K*_a_ and *P*_app_ are negative. It is not accurate to describe the intestinal absorption characteristics of realgar with the *K*_a_ and *P*_app_ values of AsIII and AsV, so the differences in absorption were analyzed with the *K*_a_ and *P*_app_ values of soluble arsenic. The *K*_a_ value of soluble arsenic in the duodenum and jejunum in realgar intestinal perfusate was higher than that in the ileum (*P* < 0.05), and there was no significant difference in *P*_app_ value of soluble arsenic in the three intestinal segments (Figure 5). The absorption rate of soluble arsenic in the duodenum in the realgar group was higher than that in the jejunum and ileum (Table 4).

When *P*_app_ < 1.8 × 10^−4^ cm/min and *P*_app_ > 1.20 × 10^−3^ cm/min of the compound in rats, the drug was defined as difficult to absorb and easy to absorb, respectively. In between, the absorptive capacity is moderate [11]. The results showed that the *P*_app_ values of soluble arsenic in realgar in the duodenum, jejunum, and ileum of rats were 5.4 × 10^−3^, 6.1 × 10^−3^, and 5.8 × 10^−3^ cm/min, respectively. It is readily absorbed in the small intestine. The gut is the main organ of absorption for oral drugs. Intestinal epithelial cells not only contain a large number of transporters that affect drug absorption but also contain many of the same metabolic enzymes as those in the liver [12]. It has been determined that human intestinal epithelial cells contain many of the same phase I and phase II metabolic enzymes as those in the liver [13]. Phase I metabolic enzymes are involved in oxidation, reduction, and hydrolysis processes. From the *C*_out_/*C*_in_ results, it can be found that AsIII in realgar is partially converted to AsV (trivalent arsenic is oxidized to pentavalent arsenic) during small intestinal perfusion. It might be that metabolic enzymes in the small intestinal epithelial cells were involved in the transformation, and the arsenic species caused an oxidation reaction. The contents of phase I metabolic enzymes in the small intestine gradually decreased with the decrease of the intestinal segment [14], so the transformation of AsIII and AsV in realgar mainly occurred in the duodenum and jejunum. Phase II metabolic enzymes in small intestinal epithelial cells mainly include glutathione-S-transferase, glucuronyl transferase, and methyltransferase enzymes [12]. They are involved in the binding reaction. Although the detected methylarsenic content is low and cannot be quantified, methylation is still found during intestinal perfusion.

### 3.4. Transmembrane Transport of Realgar in Caco-2 Cells

#### 3.4.1. Cytotoxic Effects of Drug Dissolutions in Caco-2 Cell

When realgar artificial intestinal dissolved solution group (RI) under diluting 1000 folds in Caco-2 cells, there was no significant impact on cell viability in Caco-2 cells. In detail, RI showed no cytotoxicity below the AsIII/AsV concentration of 97.1/2.5 ng/mL (Figure 6).

#### 3.4.2. Cell Transport Tests

When Caco-2 cells were incubated in a Transwell chamber for 21 days, the TEER value increased progressively and was stable above 800 Ω•cm^2^. The increase in TEER value during cell growth indicated the development of tight junctions among polarized differentiated cells. The difference of AKP between A and B sides of the Caco-2 cell monolayer was obvious, which indicated that the distribution of alkaline phosphatase was not symmetrical, and obvious polarization appeared. The above results suggest that when cells were cohesively connected and the cell monolayer was integrated, it could be used to study the mechanism of drug absorption and transport in the next step.

Caco-2 cell monolayers cultured in vitro were able to differentiate into apical (A side) and basolateral (B side) sides. The transport in the A ⟶ B direction indicates the direction of drug absorption. In fact, only the top of the intestinal epithelial cells can contact the intestinal fluid. Therefore, the mechanism of drug transmembrane transport in the A ⟶ B direction in the Caco-2 monolayer cell membrane was investigated.

The cumulative transport amount results of arsenic species are shown in Table 5. Although the accumulation of AsV in realgar decreased at 120 min, the transport of AsV through the Caco-2 cell monolayer increased with time within 180 min. This indicated that transport time was an important factor affecting the amount of arsenic species transported in Caco-2 cells, and it also suggested that arsenic species may be passively transported across the Caco-2 cell monolayer. The transmembrane transport rate of realgar was calculated based on the cumulative transport amount of soluble arsenic (Figure 7). The *P*_app_ of RI data is displayed in Table 6. The drug with complete absorption has a high permeability coefficient (*P*_app_ > 1 × 10^−6^ cm/s), and the drug with incomplete absorption has a low osmotic absorption (*P*_app_ < 1 × 10^−7^ cm/s) [15]. The *P*_app_ values of soluble arsenic for realgar in this study were higher than 1 × 10^−6^ cm/s, indicating that the soluble arsenic membrane had good permeability. As the transport time increased, the transmembrane transport rate and *P*_app_ value of soluble arsenic in realgar were increased.

### 3.5. Pharmacokinetic Study of Arsenic Species in Rat Plasma by Realgar

We quantified three arsenic species, AsIII, AsV, and DMA, in the rat. The plasma concentration-time curves of the three arsenic species are shown in Figure 8, and the main pharmacokinetic parameters are concluded in Table 7. The *C*_max_ and AUC_(0-24)_ of AsIII, AsV, and DMA in plasma of realgar were 41.26 ng L^−1^/343.977 ng h mL^−1^, 21.626 ng L^−1^/47.310 ng h mL^−1^, and 2.372 ng L^−1^/30.429 ng h mL^−1^, respectively. The order of *C*_max_ and AUC_(0-24)_ in the plasma of realgar was AsIII > AsV > DMA. AUC reflected the degree of drug absorption *in vivo,* and *C*_max_ also reflected absorption rate. The *C*_max_ and AUC of AsIII were higher than those of AsV and DMA, indicating that AsIII was most absorbed in rat plasma. *T*_max_, *t*_1/2_, and MRT_(0-∞)_ were AsV < AsIII < DMA. *T*_max_ represents the time required to reach peak drug concentration after administration. In rat plasma, AsV appeared first, followed by AsIII and DMA, which is basically the same as the metabolic sequence of arsenic reported in the study, AsV ⟶ AsIII ⟶ MMA ⟶ DMA [16]. *t*_1/2_ and MRT_(0-∞)_ reflect the average rate of drug elimination from the body and the residence time in the body, respectively. DMA is the slowest elimination in the body, and AsV elimination is the fastest, suggesting that inorganic arsenic is quickly absorbed and eliminated in the body while organic arsenic is slowly eliminated in the body.

In the 2020 edition of the Chinese Pharmacopoeia, the clinical dosage of realgar is specified at 0.05∼0.1 g. Considering factors such as arsenic metabolism and bioavailability *in vivo*, the dosage of arsenic in the rat pharmacokinetic study was 10 folds specified in the pharmacopoeia. Three arsenic compounds, AsIII, AsV, and DMA, were detected in rat plasma. Therefore, realgar bioavailability assessment using AsIII, AsV, and DMA levels is more accurate than employing total arsenic content. The change in realgar after oral administration *in vivo* is a complex process [17]. As_4_S_4_, the main component of realgar, is insoluble in water. Arsenic sulfide can be converted into soluble arsenic in an aqueous solution or gastrointestinal digestive solution. Soluble arsenic will be first dissolved in gastric fluid and exist in the form of AsIII and AsV [18]. Generally, after ingestion, arsenic is absorbed into the body in the form of AsV, then reduced to AsIII, converted to MMA and DMA through the biological methylation reaction, and finally discharged out of the body through excreta such as urine and feces [19, 20]. Arsenic metabolism usually begins with AsV, but the main component in the realgar gastrointestinal dissolution solution was AsIII. We also found that part of AsIII was converted to AsV in the small intestine, which means that the first step of inorganic arsenic metabolism is a reversible reaction. After a single oral dose, AsIII was the most absorbed component of the arsenic species in rat plasma. Studies have shown that after the oral administration of realgar for 30 days, DMA is the component with the highest arsenic content in rats [21]. We speculated the reason may be that the methylation of inorganic arsenic takes a period of time and is a process in vivo. After a single administration, taking the plasma several times in a short period of time affected the content of inorganic arsenic in the plasma, resulting in a decrease in the degree of methylation and a decrease in the content of DMA.

## 4. Conclusions

This study analyzed the arsenic species to explore the absorption process of arsenic in realgar. Realgar absorption assessment of AsIII, AsV, and DMA levels was more accurate than employing total arsenic content in this study. Realgar could convert into soluble arsenic in gastrointestinal digestive solution. Soluble arsenic was first dissolved in a gastrointestinal fluid and existed in the form of AsIII and AsV, and it was further methylated to MMA and DMA. Arsenic metabolism usually begins with AsV, but a part of AsIII could be converted to AsV in the small intestine in this study. It has been suggested that the first step of inorganic arsenic metabolism may be a reversible reaction.

## Figures and Tables

**Figure 1:** Reductive-oxidative methylation metabolic pathway of arsenic. AsV is first reduced to AsIII under the action of glutathione (GSH). AsIII is converted to MMAV after catalysis by methyltransferase (AS3MT), at the same time S-adenosylmethionine (SAM) and GSH providing methyl donors. MMAV is converted to MMAIII under the action of GSH, and MMAIII is secondary methylated to DMAV under the action of AS3MT, SAM, and GSH.

**Figure 2:** Chemical structures of six arsenic species.

**Figure 3:** Cumulative dissolution-time curves of AsIII, AsV, and soluble arsenic in artificial gastric fluid (a) and artificial intestinal fluid (b) with realgar (*n* = 3).

**Figure 4:** Comparison of cumulative dissolution of AsIII (a), AsV (b), and soluble arsenic (c) in realgar in artificial gastrointestinal fluid (*n* = 3), compared with the artificial gastric fluid group (^*∗*^*P* < 0.05).

**Figure 5:** *K*_a_ and *P*_app_ results of arsenic species in realgar intestinal perfusate in different intestinal segments of rats (*n* = 6), compared with soluble arsenic duodenum, (^*∗*^*P* < 0.05).

**Figure 6:** Cytotoxicity tests of drug dissolution solution as performed by the MTT assay in Caco-2 cells. Cell viability of Caco-2 cells was exposed to a series of concentrations of realgar artificial intestinal dissolved solution. (*n* = 6). ^*∗*^Denoted results are significantly different from the control group, (*P* < 0.05).

**Figure 7:** Transmembrane transport rate of soluble arsenic in realgar artificial intestinal dissolved solution in the Caco-2 cell model (A ⟶ B), (*n* = 3).

**Figure 8:** Mean plasma concentration-time curves of the AsIII (a), AsV (b), and DMA (c) after administrating 0.1 g/kg realgar (*n* = 6).

**Table 1:** Chromatographic parameters of HPLC-ICP-MS.

Time (min)	A (%)	B (%)
0∼15	0 ⟶ 100	100 ⟶ 0
15∼20	100 ⟶ 0	0 ⟶ 100
20∼25	0	100

**Table 2:** Cumulative dissolution rate of soluble arsenic from realgar in artificial gastrointestinal fluid.

Time (*h*)	Artificial gastric fluid	Artificial intestinal fluid
1	6.92%	—
2	15.72%	38.19%
4	21.99%	45.70%
6	—	52.16%
8	—	59.20%

**Table 3:** *C*_out_/*C*_in_ results of arsenic species in realgar intestinal perfusate at different intestinal segments and at different times (*n* = 6, Mean ± SD).

Intestinal segment	Time (*h*)	C_out_/C_in_		
		AsIII	AsV	Soluble arsenic
Duodenum	15	0.26 ± 0.21	3.14 ± 0.81	0.73 ± 0.04
	30	0.29 ± 0.20	3.16 ± 0.91	0.75 ± 0.04
	45	0.32 ± 0.16	3.01 ± 0.96	0.77 ± 0.02
	60	0.30 ± 0.25	3.20 ± 1.04	0.77 ± 0.03
	75	0.33 ± 0.24	3.17 ± 0.86	0.79 ± 0.03

Jejunum	15	0.59 ± 0.10	1.54 ± 0.46	0.76 ± 0.06
	30	0.62 ± 0.10	1.46 ± 0.39	0.77 ± 0.06
	45	0.63 ± 0.12	1.50 ± 0.28	0.79 ± 0.08
	60	0.67 ± 0.09	1.34 ± 0.25	0.79 ± 0.06
	75	0.70 ± 0.08	1.28 ± 0.24	0.80 ± 0.06

Ileum	15	0.84 ± 0.05	0.78 ± 0.11	0.80 ± 0.08
	30	0.85 ± 0.06	0.77 ± 0.10	0.80 ± 0.07
	45	0.86 ± 0.07	0.76 ± 0.12	0.82 ± 0.08
	60	0.86 ± 0.06	0.78 ± 0.11	0.82 ± 0.07
	75	0.86 ± 0.05	0.80 ± 0.13	0.83 ± 0.06

**Table 4:** Absorption rate of soluble arsenic in realgar in the small intestine (*n* = 6, Mean ± SD).

Intestinal segment	Absorption rate (%)
Duodenum	24.69 ± 3.97
Jejunum	20.30 ± 6.83
Ileum	17.21 ± 7.77

**Table 5:** Cumulative transport amount in A ⟶ B of realgar artificial intestinal dissolved solution in Caco-2 cells (*n* = 3, Mean ± SD).

Time (min)	Cumulative transport amount (*n*g)		
	AsIII	AsV	Soluble arsenic
30	6.26 ± 1.21	0.23 ± 0.07	6.49 ± 1.05
60	11.66 ± 0.92	0.41 ± 0.06	12.06 ± 0.97
90	16.95 ± 0.57	1.01 ± 0.16	17.96 ± 0.55
120	21.97 ± 0.44	0.84 ± 0.02	22.81 ± 0.46
180	29.84 ± 1.26	1.20 ± 0.15	31.04 ± 1.18

**Table 6:** Apparent permeability coefficients (*P*_app_) in A ⟶ B of realgar artificial intestinal dissolved solution in Caco-2 cells (*n* = 3, Mean ± SD).

Time (min)	*P*_app_ (cm/s)
30	3.23 × 10^−5^ ± 5.22 × 10^−6^
60	6.01 × 10^−5^ ± 4.84 × 10^−6^
90	8.95 × 10^−5^ ± 2.76 × 10^−6^
120	1.14 × 10^−4^ ± 2.30 × 10^−6^
180	1.55 × 10^−4^ ± 5.90 × 10^−6^

**Table 7:** Pharmacokinetic parameters of AsIII, AsV, and DMA after administrating realgar.

Parameter	Unit	AsIII	AsV	DMA
*T*_max_	*h*	2.571	0.393	3.143
*C*_max_	ng·L^−1^	41.26	21.626	2.372
AUC_(0-24)_	ng·h·mL^−1^	343.977	47.310	30.429
AUC_(0-∞)_	ng·h·mL^−1^	369.762	47.687	42.014
*t*_1/2_	*h*	5.45	1.775	11.273
MRT_(0-∞)_	*h*	9.649	2.790	23.145

## Data Availability

The data used to support the findings of this study are available from the corresponding author upon request.

## Abbreviations

AsIII: Arsenite
AsV: Arsenate
AsB: Arsenobetaine
AsC: Arsenocholine
AUC: The area under the concentration-time curve
AS3MT: Arsenite methyltransferase
As_4_S_4_: Tetra-arsenic tetrasulfide
*C*_max_: The peak concentration
DMA: Dimethylarsonic acid
DMAIII: Dimethylarsonous acid
GST: Glutathione s-transferases
HPLC-ICP-MS: High-performance liquid chromatography-inductively coupled plasma-mass spectrometry
*K*_a_: Absorption rate constant
LLOQ: Lower limit of quantitation
MMA: Monomethylarsonic acid
MRT: Average residence time
MMAIII: Monomethylarsonous acid
*P*_app_: The apparent permeability coefficients
QC: Quality control
*T*_max_: The peak time
*T*_1/2_: The terminal elimination half-life
TEER: Transepithelial electrical resistance.
